This article has been retracted.

# Prevention Methods of Fitness and Bodybuilding Exercise Injury Based on Data Mining

**DOI:** 10.1155/2022/7083991

**Published:** 2022-04-14

**Authors:** Jun Xie

**Affiliations:** School of Physical Education and Health, A'ba Teachers' University, Wenchuan, 623002 Sichuan, China

## Abstract

Fitness and bodybuilding are becoming the trend of the development of sports projects today, not only to bring health to the exercisers, but also to keep the body in good condition. However, due to the wrong attitudes and methods of exercisers, they often have negative effects on exercisers, such as sprains, strains, and tendon strains. This article is based on data mining technology to realize the research of exercise injury prevention methods, so firstly, it introduces the steps and applications of data mining technology and highlights the cluster analysis method in data mining technology. Then it discusses the injury factors of fitness and bodybuilding and outlines the best measures to prevent exercise injury. At the same time, the C4.5 algorithm was introduced to realize the processing of the data set, and the effectiveness of preventive measures was proved by investigating the damage of fitness and bodybuilding exercises in 15 clubs in a certain city. The results of the study show that the number of people who exercise more than 3 times a week accounts for 65.6% of the total number of people, which shows that exercisers in a city's fitness club exercise more frequently each week.

## 1. Introduction

The society is developing rapidly, and the nationwide fitness program is being implemented more and more. Most sports enthusiasts agree to spend money on exercise. However, from the perspective of long-term training goals, many bodybuilders are injured, which has some negative effects on bodybuilders who want to continue training during actual exercise. Therefore, it is very important to take appropriate and timely treatment measures and methods, and we must attach great importance to the prevention of sports and sports injuries. Only by strengthening the awareness of exercise injury prevention can the occurrence of injury be avoided as much as possible.

Regarding the research on data mining and fitness exercise injury prevention methods, scholars at home and abroad have provided a large number of references. Amodio uses the People-Environment-Occupation (P-E-O) framework to determine the factors that cause traumatic brain injury in male and female workers. The study found five factors: unexplained human factors, colleagues' behavior, external environment, safety measures, and equipment failures. Due to equipment failure or malfunction, male workers are more likely to experience traumatic brain injury than female workers. A statistically significant gender difference was observed in the P-E-O factor [1]. Cui researched data mining based on intelligent recommendation system. First, mathematically model the intelligent recommendation system based on association rules. Then, the fuzzy clustering algorithm is used to optimize the system. After the system is built, the performance of the system is evaluated. The evaluation indicators include accuracy, coverage, and response time. Finally, put the system into trial operation on the e-commerce platform. Comparing the click-through rate and purchase conversion rate of recommended products before and after operation, randomly launch a questionnaire survey to platform users to analyze user satisfaction [2]. Shin found that classification, text mining, and clustering are the main data mining techniques used by researchers. Compared with the field of mathematics education, the research using data mining is more likely to be carried out in the field of science education. Shin provides enlightenment for the research and teaching of science and mathematics and proposes potential research directions [3]. Bbosa compared parametric techniques in the form of naive Bayes and logistic regression with non-parametric techniques in the form of support vector machines and artificial neural networks to determine which model is best for predicting the unbalanced malaria incidence data set [4]. Based on experimental data obtained under various environmental settings, Zhao C analyzed the probability distribution of skin reflection model parameters in RGB space. Based on this distribution, a new pulse extraction algorithm is proposed, which uses the center of the distribution as a model parameter for preliminary pulse separation and uses a cascaded minimum mean square adaptive filter to compensate the modeling error [5]. Min briefly emphasized the positive effects of exercise on promoting brain function. In general, Min provides an understanding of the importance of motor neuroscience and emphasizes recommendations for future health research [6]. The data of these studies are not comprehensive, and the experimental conclusions are yet to be discussed, so they cannot be popularized and cannot be recognized by the public.

The innovation of this research is to use the cluster analysis method of data mining technology, combined with the C4.5 algorithm to realize the research of exercise injury prevention methods. In this way, not only can the knowledge that is useful for the core of the research be extracted, but also some methods that have never appeared can be integrated and analyzed based on this knowledge. In addition, this research has collected data in the field of fitness and bodybuilding by means of investigation, which shows the effectiveness and robustness of the research. Finally, it expounds the factors of fitness and fitness exercise injury from the four aspects of physiology, psychology, technology, and clubs and comprehensively summarizes the injury prevention methods.

## 2. Data Mining Technology and Fitness and Bodybuilding Exercise Injury Prevention

### 2.1. Data Mining

Data mining is the process of extracting potentially useful information and knowledge hidden in it that people do not know beforehand from a large amount of incomplete, noisy, fuzzy, and random data.

The use of data mining technology is inseparable from the data warehouse, so here is a brief introduction to the structure of the data warehouse, as shown in Figure 1.

Data mining includes the following steps, as shown in Figure 2:

1. It obtains data for analysis [7]. Data mining resources can take many forms, but to create a good model, it must have a high-quality information source. The data in the database system is filtered and cleaned with high-quality information. Therefore, obtaining the source from the database is a wise choice
2. It chooses appropriate data processing tools and algorithms for data mining [8, 9].
3. It explains the results. Since the results of data mining do not provide a direct explanation for a specific field, it is very important for relevant personnel to analyze the results to determine the success or failure of the data mining project [10]. If the data extraction results are not satisfactory, the reasons should be analyzed and reused
4. It applies the results to the problem to be solved. Data mining is a repetitive process. In the repetitive process, it tends to be more towards the essence of things [11].

The general processing flow of data mining is clear goals, data preparation, model building, evaluation and interpretation of output results, and implementation of 5 stages. The processing flow is shown in Figure 3 [12].

#### 2.1.1. Clear Goals

The main task of a data mining application is to locate and explain the problems that need to be solved. In addition to choosing a suitable extraction method, the target details should also be detailed and clear in order to study the impact of data extraction and the effectiveness of the model creation [13].

#### 2.1.2. Data Preparation

It extracts the required data according to the purpose of the data mining business. In addition to necessary checks and corrections to ensure data quality, data compatibility between different sources should also be considered. If there are multiple data fields in the data set, it should use a specific method to find the data field that has the greatest impact on the model output and reduce the input fields accordingly. Commonly used methods are “descriptive data mining” and link analysis. Combining multiple variables (addition, subtraction, ratio, etc.) may have a greater impact than these variables. If expand the scope of certain variables, then these variables are very good predictors. Therefore, it is necessary to consider whether to create some new variables during the data preparation process. Dealing with missing data is also an important part of the data preparation process, some of which are very important in themselves [14, 15].

#### 2.1.3. Building a Model

Building a model is the most important step in the entire data mining process. It serves as the basis of data mining. Whether the model is built or not will determine whether the output results meet the requirements [16].

#### 2.1.4. Evaluation and Interpretation of Output Results

After the model is created, its effectiveness must be evaluated and its value explained. For practical applications, the model validity criteria will vary depending on the application data. However, accuracy is not the only way to evaluate the best design. The analysis of the results should take into account the type of error and related cost factors. If the cost of each calculation error is different, the lowest cost model (not necessarily the smallest error) will be a better choice. It is important to test the model directly from actual needs and solve actual problems. First apply in a small area and then gradually expand the coverage area until sufficient test results are obtained [17].

#### 2.1.5. Implementation

After creating and verifying the template, there are two main ways to use it. One is to allow relevant personnel to analyze and make comments and suggestions; the other is to use templates for different data sets. This model can be used to determine the type of case, or it can be used in other databases to select records that meet specific needs, so that tools can be used for further analysis. After applying the model, it need to continuously monitor the effectiveness of the model. Even if the model is used successfully, the tracking cannot be undone. This is because things are constantly evolving, and when the unit's requirements, capabilities, and conditions change over time, the model may no longer be effective. Therefore, as the time spent on the model increases, new models need to be continuously tested, and sometimes new models are created [18].

In a nutshell, the data mining process generally consists of three main stages: data preparation, mining operations, result expression, and interpretation.

*(1) Data Preparation Process*. This process can be divided into three subphases: data integration, data selection, and preprocessing. Data integration is to integrate data into a multi-file or multi-database operating environment to solve semantic instability, manage data instances, and clean up dirty data. The purpose of data selection is to identify the data set that needs to be analyzed, reduce processing boundaries, and improve the quality of data extraction. Data preprocessing is to overcome the limitations of current data mining tools.

*(2) Data Mining Stage*. In this stage, actual mining operations are carried out. The key points included are the following:

1. First decide how to generate hypotheses, whether to let the data mining system generate hypotheses for users or whether users themselves make hypotheses about the knowledge that may be contained in the database. The former is called discovery data mining, and the latter is called verification data mining
2. Choosing the right tool
3. The operation of mining knowledge
4. Confirming the discovered knowledge

*(3) Result Presentation and Interpretation Stage*. Analyze the extracted information according to the decision-making purpose of the end user, distinguish the most valuable information, and submit it to the decision-maker through decision support tools. Therefore, the task of this step is not only to express the results, such as the use of information visualization methods, but also to filter the information.

Cluster analysis is a commonly used method of data mining. There are various methods of cluster analysis. The more commonly used methods can be simply summarized as follows:

*(1) Clustering Method Based on Partition*. The total number of clusters K that is less than the number of objects in the data set is preset, and the division is performed on this condition, and finally K clusters are obtained. These K groups meet the following conditions: at least one piece of data belongs to each group, and for each piece of data, it can only belong to a specific group and cannot appear in multiple different groups at the same time. The execution of the algorithm can be seen as an iterative process. First, the data is divided into K groups according to the K value, and then after result evaluation and iterative methods, each time the attribution of the data in the group is corrected, after the process converges, a clustering result is obtained [19].

*(2) Hierarchical Clustering Method*. The hierarchical clustering method first initializes a clustering tree and then decomposes the data according to the hierarchical relationship between the data until the preset conditions are met. On the one hand, due to the different actual situations that need to be dealt with, and on the other hand, considering the needs of algorithm implementation, the order of hierarchical clustering can be divided into (1) top-down and (2) bottom-up [20].

*(3) Density-Based Clustering Method*. The clustering method based on distance measurement is largely limited by the distance definition method and can only mine simple clusters with a relatively regular shape (spherical). In response to this shortcoming, some scholars have proposed a density-based clustering method, which uses the density of data to construct clusters and can produce clustering results of arbitrary shapes. The method is specifically described as analyzing the tightness between the data and presetting a density threshold; when the density of the data is higher than this threshold, the data points in the area are gathered into clusters. At the same time, compared with the distance measurement method, this method is not affected by the noise of outliers to a greater extent and obtains better results [21].

*(4) Model-Based Clustering Method*. This method deeply studies the existing model and analyzes the data characteristics of the data set to be mined on the basis of it, so that the subdata set consistent with the model characteristics is regarded as a cluster. Before the clustering starts, the model is specified according to the characteristics of the data set, and the data conforming to the model is gathered into clusters to form clusters [22]. One of its underlying assumptions is that the generation of the data set to be mined conforms to a certain probability density distribution. In this type of algorithm, the clustered data is also automatically determined based on statistics, and noise and outliers are also analyzed through statistics [23].

There is also a commonly used data mining method—association rules. The core purpose of association rule analysis is to discover the interrelated and interdependent relationships that exist in the data. Association rule mining is also a data mining method derived from database theory and has a very wide range of practical applications. Specifically, in relational databases, there are often some data that appear synchronously, which is called a pattern. When this pattern appears frequently in the database, it is considered that there is a specific association relationship, which is called an association rule.

The architecture of data mining is shown in Figure 4:

An authoritative survey report pointed out that data mining technology will develop rapidly within 3-5 years and be widely used in all walks of life. The development of technology is always driven by the increase in demand. Due to the great development of the information industry, various fields and industries have begun their informatization construction, which has caused an explosive growth in the scale of data, and massive data cannot be left unused as data. Data mining methods can find relevant knowledge that is useful to humans and can improve the efficiency of production and life from these massive data and use this knowledge to further promote the rapid and steady development of productivity. It is precisely because of this that the research of data mining technology has become the current research hotspot in the field of database, machine learning, and statistics, and various rich application examples have been completed.

The application of data mining is extremely wide. Through the combination of specific data in various industries and fields, many professional data mining basic applications have been produced, representative of which are applications in the retail industry, insurance industry, astronomical and meteorological research, food engineering, and biotechnology.

Compared with the above majors, data mining technology is used more widely in the business field, and the more typical applications are marketing and shopping basket analysis. The former conducts basic clustering of customers through the mining and analysis of user historical purchase data and distinguishes key customers from general customers. Selectively increasing marketing efforts for key customers can effectively improve marketing effects. The latter is mainly used in retail industries such as supermarkets, through massive retail data, to refine the buying habits of shoppers, in order to adjust the way the goods are placed. While providing customers with a convenient shopping environment, it has also increased the actual operating income of the supermarket. One of the representative examples is the successful case of “Beer and Diapers.”

In addition, data mining has a very wide range of applications in the banking and financial industries, such as risk assessment and price prediction.

### 2.2. Fitness and Bodybuilding Exercise Damage Prevention

According to different analysis angles, the classification of exercise injuries can be roughly divided into the following categories:

1. According to the damaged tissue, it can be divided into muscle injury, ligament injury, nerve injury, blood vessel injury, bursal injury, tendon sheath injury, cartilage injury, etc.
2. According to the severity, it is divided into severe injury, moderate injury, and mild injury
3. Severe injury. Cannot exercise at all for more than one week after injury and needs rest and treatment
4. Moderate injury. The normal physical exercise cannot be carried out according to the training plan within one week after the injury, and local physical activities need to be stopped or reduced
5. Mild injury. After injury, normal training can be carried out in accordance with the teaching and training plan, and the injury will not be aggravated
6. According to the integrity of the skin and mucous membrane after sports injury, it can be divided into: closed injury and open injury
7. Closed injury. The skin and mucous membrane of the injured area remain intact, with no cracks communicating with the body surface
8. Open injury. The skin or mucous membrane of the injured area is destroyed, and there are cracks communicating with the body surface

#### 2.2.1. Injury Factors

*(1) Technical Factors*. *(1) Incorrect Technical Action*. Most of the injuries caused by incorrect technical movements are aimed at beginners. Due to the wide variety of exercises during the exercise, it is difficult to master technical activities in a short period of time. However, out of curiosity, beginners often prefer new exercises. Studies have shown that most beginners do not actively learn fitness knowledge and are seriously lacking in science. In terms of fitness equipment, most beginners imitate the movements of European and American bodybuilders through online videos and take some methods that are not suitable for beginners to complete technical movements. For exercisers, mastering the correct exercise technique is a reliable way to improve their fitness performance while avoiding injuries caused by technical exercise errors.

*(2) Violation of the Principle of Gradual and Orderly Progress*. The complexity of sports training should be based on the principle of combining practice from simple to heavy and from simple to visual. Under the influence of external conditions, the body gradually adapts and produces repeated stimulation. Therefore, it is impossible to change the shape, function, physical activity, and other adaptive changes of various organs and systems of the body through high-intensity training. Instead, repeated training creates a gradual process of adaptation. The health of the human body is a process of gradual accumulation. Excessive exercise not only fails to obtain the effect of exercise, but also leads to sports injuries. In the early stages of exercise, beginners may blindly perform high-intensity exercise without mastering the correct and necessary exercise skills, resulting in incorrect exercise movements and impaired physical function.

*(3) Partial Load Is Too Heavy*. The dynamic changes of load play an important role in the development of exercise posture, improvement of physical fitness, and load management within the range of physical endurance capabilities. It is of great significance to improve the sports ability of members and prevent sports injuries. The scientific nature of training is to know how much exercise the body can or should take, and adjust to own physical condition in time, rather than causing deformity or injury. Therefore, exercisers should consider their own physical characteristics during the training process to reduce the injury rate.

*(4) Unreasonable Warm-Up Activities*. Unreasonable warm-up activities mainly include insufficient warm-up activities, excessive warm-up activities, failure to do warm-up activities, unreasonable connection between activity content and training content, and excessive time between warm-up activities and formal training or competition.

*(2) Physiological Factors*. *(1) Poor Physical Fitness*. Physical fitness is usually a comprehensive manifestation of the functions of various organs and system muscles in the human body. Physical fitness usually includes speed, strength, endurance, agility, and flexibility. Good exercise is not only an important basis for improving the ability of exercisers, but also an important guarantee for preventing sports injuries and reducing the degree of injury.

*(2) Body Fatigue*. Sports fatigue is the reduction of physical strength during exercise. After a good rest, the body's functions can be restored. The principle of improving physical function through training is not only stress-fatigue-relieving fatigue-recovery. Therefore, scientifically and optimally adjusting the recovery speed of each load can make training more effective. When physical fatigue cannot be recovered in time and effectively, exercise performance is poor, such as poor exercise coordination, decreased strength, and technical dyskinesias during exercise. Exercisers after get off work should be based on their own feelings rather than training plans. Stop the training when feel tired; when full of energy, increase the training intensity accordingly.

*(3) Psychological Factors*. *(1) Inattention*. Studies have shown that it is difficult for people to maintain long-term concentration, which is also a normal phenomenon. People's attention is easily distracted by changes in the outside world and also changes due to changes in their own emotions. There are roughly several reasons for inattention: fatigue, environment, psychology, etc. When people exercise when they are inattentive, their reaction speed will slow down. Therefore, it should develop the habit of concentration during daily training or can exercise some training to exercise the problem of concentration, so as to slowly form a set of training framework for own concentration and avoid injury caused by inattention.

*(2) The Training Mood Is Too Excited or Low*. When a person's emotions are too excited or low during training, some physical injuries often occur. For example, lifting a barbell when too excited may cause to exceed usual training volume due to emotional reasons. If the individual did not pay attention at the time, this will cause hand injuries. And in the case of too low, it is very likely that the whole body will be ignored due to one's own emotional reasons, which is also very prone to injury.

*(4) Fitness Club Factors*. *(1) Poor Venue*. There are some projects that cannot be separated from a good venue. Aerobics, for example, involves some jumping movements, so if the venue is too hard, slippery, or unequal, it will affect the progress of the training program and cause damage to the human body.

*(2) Device Factors*. The damage caused by equipment factors mainly includes the following situations: equipment aging, lack of maintenance, warning signs indicating defects, and unreasonable design. Some surveys show that the more serious one is the injury caused by the treadmill, which is mainly because the speed is set too fast. In addition, loose screws, high friction, and inconsistent left and right weights may cause damage. In this case, it is necessary for the club to do regular inspections and maintenance, and the exercisers themselves must carefully check the condition of the equipment before using the equipment.

#### 2.2.2. Countermeasures to Prevent Exercise Injury

People pay more attention to the improvement of their own comprehensive quality. The number of people participating in fitness and bodybuilding exercises continues to increase. The intensity and density of exercises increase accordingly, and the chances of injury are also increasing. Preventive measures become more important.

*(1) Strengthen Ideological Education and Theoretical Guidance and Improve Exercisers' Awareness of Preventing Exercise Injuries*. The core reason for the higher injury rate is the lack of awareness of self-protection of exercisers and the lack of awareness of preventing exercise injury. Therefore, it is necessary for exercisers to strengthen the study of the basic theoretical knowledge of exercise injuries and improve their awareness of prevention and the ability to deal with injuries according to the actual situation, so as to treat exercise injuries correctly.

*(2) Reasonably Arrange Training Content and Load*. The content and load of training should be arranged according to the individual's own situation. If high-load training is carried out due to impulse or other motivations, it will cause personal injury. Therefore, it is particularly important to arrange the content and load of training reasonably. At the same time, adjust the arrangement in time according to own situation, so as to avoid physical damage as much as possible.

*(3) Pay Attention to Comprehensive Training of Physical Fitness*. The original intention of exercise is to have a strong physique. Therefore, in actual training, attention should be paid to the overall improvement of physical fitness, so as to prevent the occurrence of exercise injuries.

*(4) Checking the Equipment*. Develop the habit of checking whether the equipment is broken and firm every time you start exercising, so that it can also avoid exercise damage due to equipment problems.

When an exerciser is injured, he should first determine whether his condition is critical. If the situation is critical, he should call for help immediately; if there is no major problem, he should deal with it by himself or go to the hospital for examination.

## 3. C4.5 Algorithm

The classification rules generated by the C4.5 algorithm are easy to understand and have a high accuracy rate. The C4.5 algorithm uses the information gain rate to optimize the attributes of the decision tree, and the information gain rate calculation method is as follows:

Supposing a data set *T*, a classification set {*C*_1_, *C*_2_, *C*_3_ ⋯ *C*_*k*_}, and the data set *T* is divided into multiple subsets by the attribute *V*. Supposing that *V* has *n* values {*v*_1_, *v*_2_, *v*_3_ ⋯ *v*_*n*_}, and each value is not repeated. The data set *T* is divided into *T*_1_, *T*_2_, *T*_3_ ⋯ *T*_*n*_, and the value of all instances in *T*_*i*_ is *v*_*i*_.

Probability of category occurrence:

(1) $$\begin{array}{c} P\left(C_{j}\right)=\left|C_{j}\right|/\left|T\right|=freq\left(C_{j},T\right)/\left|T\right|. \end{array}$$

Probability of attribute:

(2) $$\begin{array}{c} P\left(v_{i}\right)=\left|T_{i}\right|/\left|T\right|. \end{array}$$

In the attribute instance, the conditional probability of class *C*_*j*_:

(3) $$\begin{array}{c} P\left(C_{j}\left|v_{j}\right.\right)=\left|C_{jV}\right|/\left|T_{i}\right|. \end{array}$$

Information entropy of category:

(4) $$\begin{array}{c} H\left(C\right)=-\underset{j}{\sum }P\left(C_{j}\right)\log_{2}\left(P\left(C_{j}\right)\right)=-\underset{j}{\sum }\frac{freq\left(C_{j},T\right)}{\left|T\right|}*\log_{2}\left(\frac{freq\left(C_{j},T\right)}{\left|T\right|}\right)=\inf o\left(T\right). \end{array}$$

The conditional entropy of the category divides the set *T* according to the attribute *V*, and the conditional entropy of the category after segmentation:

(5) $$\begin{array}{c} H\left(C\left|V\right.\right)=-\sum P\left(v_{i}\right)\sum P\left(C_{j}\left|v_{j}\right.\right)\log_{2}\left(P\left(C_{j}\left|v_{i}\right.\right)\right)=\overset{n}{\underset{i=1}{\sum }}\frac{\left|T_{i}\right|}{\left|T\right|}*\inf o\left(T_{i}\right)=\inf ov\left(T\right). \end{array}$$

Information gain:

(6) $$\begin{array}{c} I\left(C,V\right)=H\left(C\right)-H\left(C\left|V\right.\right)=\mathrm{int}o\left(T\right)-\inf ov\left(T\right)=gain\left(V\right). \end{array}$$

Information entropy of attribute *V*:

(7) $$\begin{array}{c} H\left(V\right)=\underset{i}{\sum }p\left(v_{i}\right)\log_{2}\left(P\left(v_{i}\right)\right)=-\overset{n}{\underset{i=1}{\sum }}\frac{\left|T_{i}\right|}{\left|T\right|}*\log_{2}\left(\frac{\left|T_{i}\right|}{\left|T\right|}\right)=spit\_\inf o\left(V\right). \end{array}$$

Information gain calculation formula:

(8) $$\begin{array}{c} gain\_ratio=gain\left(V\right)/spit\_\inf o\left(V\right). \end{array}$$

Relationship coefficient:

(9) $$\begin{array}{c} \Delta \min=\underset{i}{\min}\underset{k}{\min}\left|y_{0}\left(k\right)y_{i}\left(k\right)\right|, \end{array}$$

(10) $$\begin{array}{c} \Delta \max=\underset{i}{\max}\underset{k}{\max}\left|y_{0}\left(k\right)y_{i}\left(k\right)\right|, \end{array}$$

(11) $$\begin{array}{c} \Delta =\left|y_{0}\left(k\right)-y_{i}\left(k\right)\right|, \end{array}$$

(12) $$\begin{array}{c} \xi_{i}\left(k\right)=\frac{\Delta \min+\alpha \Delta \max}{\Delta +\alpha \Delta \max}. \end{array}$$

Grey correlation calculation:

(13) $$\begin{array}{c} f_{i}=\frac{1}{m}\overset{m}{\underset{k=1}{\sum }}\xi_{i}\left(k\right). \end{array}$$

Net input of unit *j*:

(14) $$\begin{array}{c} I_{j}=\underset{i}{\sum }w_{ij}O_{i}+\theta_{j}. \end{array}$$

Error Err_j_ of output layer unit *j*:

(15) $$\begin{array}{c} E{\text{rr}}_{j}=O_{j}\left(1-O_{j}\right)\left(T_{j}-O_{j}\right). \end{array}$$

Error of hidden layer unit *j*:

(16) $$\begin{array}{c} E{\text{rr}}_{j}=O_{j}\left(1-O_{j}\right)\underset{k}{\sum }{Err}_{k}w_{kj}. \end{array}$$

Weight update:

(17) $$\begin{array}{c} \omega \left(k\right)=\omega \left(k-1\right)+\Delta \omega \left(k\right)+a\omega \left[\left(k-1\right)-\left(k-2\right)\right]. \end{array}$$

Z-score like formula:

(18) $$\begin{array}{c} v^{\prime }=\frac{v-\overset{—}{A}}{\sigma_{A}}. \end{array}$$

Min–max normalized conversion function:

(19) $$\begin{array}{c} v^{\prime }=\frac{\text{x}-\min}{\max-\min}. \end{array}$$

The number of hidden layer nodes can be determined by experimental methods:

(20) $$\begin{array}{c} \text{b}=\sqrt{m+n}+a. \end{array}$$

Among them, a is a constant between 0 and 10, *m* is the number of nodes in the output layer, and *n* is the number of nodes in the input layer.

Through the method of quantitative and qualitative evaluation of the structure and content of the questionnaire, relevant experts are asked to evaluate the content indicators of the questionnaire according to five levels: *A* is very suitable, *B* is more suitable, *C* is general, *D* is general suitable, and E is not suitable. The specific evaluation results are shown in Table 1:

Taking 18-60 year-old people from 15 fitness clubs in 8 districts of a city as the research object, we randomly sampled 20 people from each club, half of them male and female. Among the 275 valid questionnaires returned, 85 people have experienced exercise injuries, with a total of 120 injuries.  Figure 5 shows the statistics of the number of injured male and female ratios.

It can be seen from Figure 5 that the proportion of male injuries is 57.6%, which is slightly higher than the 42.4% of females. There is no statistically significant difference between the two. Among the secondary and above injuries, 88.6% of men were significantly higher than 11.4% of women, and there was a significant difference between the two.

Investigating the relationship between people's fitness orientation and motivation and exercise injury, it is found that fitness motivation generally includes health, relieving work pressure, reducing fat and shaping, and increasing muscle content as shown in Table 2.

It can be seen from Table 2 that the proportion of different motivational injuries is different. Women's pursuit of appearance is much higher than that of men. They tend to lose fat and shape their bodies. They are keen on aerobics, yoga, and other body exercises and various jumping exercises. They have more exercises. The main motivation of men is to increase muscle content and relieve work pressure, and they are keen on fitness equipment.

The main types of knee injuries include sprains, lacerations, and strains, as shown in Table 3. An example of knee injury is shown in Figure 6.

In fitness club knee exercise injuries, the main manifestations are men, and they are mainly caused by training factors, such as heavy squats and leg lifts, followed by long-term exercises, and overloaded spinning exercises. Knee joint injuries are mostly caused by exercisers' incorrect technical movements, large movements, repeated overloading of the knee joints, and sports fatigue.

The waist sports injuries of exercisers in fitness clubs are mostly acute injuries. The nature and proportion of waist injuries are shown in Table 4. An example of waist injury is shown in Figure 7.

There are many reasons why exercisers may cause sports injuries during exercise. In order to find out the main injury factors and analyze them in detail, a questionnaire for sports injury factors for exercisers in fitness clubs is designed; 10 injury factors were determined, and after statistical analysis, the results are shown in Table 5.

According to the investigation and statistics of the injury site, it is found that the incidence of ankle joint injury is the highest, and it is mainly concentrated in women, as shown in Figure 8.

It can be seen from Figure 8 that the injured parts of male exercisers are relatively scattered, while the injured parts of females are mainly concentrated in the lower extremities.

Whether male or female, the most vulnerable tissues are ligaments, tendons, and muscles, as shown in Figure 9.

It can be seen from Figure 9 that compared with the female exercise group, the male exercise group is more prone to damage to ligaments, tendons, and muscles.

The relationship between fitness years of exercisers and sports injuries is shown in Figure 10(a). The relationship between exerciser's fitness frequency and sports injury is shown in Figure 10(b).

It can be seen from Figure 10(a) that most exercisers lack common sense of fitness, have poor physical fitness, and are prone to sports injuries. With the increase in fitness years, the injury rate gradually decreases, which has a certain relationship with the improvement of exercisers' physical fitness, the increase of fitness knowledge, and the enhancement of fitness experience. From Figure 10(b), it can be seen that the number of people who exercise more than 3 times per week accounted for 65.6% of the total number of people, which indicates that exercisers in a fitness club in a city have a higher number of exercises per week

## 4. Discussion

With the increasing popularity of sports and bodybuilding, many bodybuilding enthusiasts like to do simple exercises, hoping to have a strong body. The goal of exercisers is to change from simple participation to gradual improvement in body shape. However, exercise is often accompanied by injuries during exercise, which may be dangerous to the athlete's body and will significantly reduce their enthusiasm for exercise.

Sports injury is an injury that occurs in sports activities, and the injured part is closely related to sports equipment and sports equipment. Related research results show that compared with other parts of the body, limb joints are more prone to limb injuries during exercise. Due to the large number of joints, the external force is quite large, leading to various injuries during exercise. Many injuries occur during sports, such as running and swimming.

Data mining technology can analyze and learn patterns and rules useful to users from a large amount of data. Using these learned patterns and rules, when new sample data is available, the possible characteristics of the sample data can be predicted based on the existing patterns and rules.

## 5. Conclusion

Exercise has a positive effect on physical and mental development, but if the movement is not standard or the preparation before exercise is not sufficient, it is easy to cause injury. Therefore, we must be highly vigilant about sports safety and be fully prepared before exercise to prevent injuries. This article mainly explains the injuries that are likely to occur in fitness exercises, do a good job in the prevention of sports injuries, reduce the incidence of injuries, and do better exercises while ensuring that the body is not damaged. This article analyzes the injuries that are likely to occur in the process of fitness exercise and puts forward some reasonable suggestions.

## Figures and Tables

**Figure 1:** Data warehouse architecture.

**Figure 2:** The process of data mining.

**Figure 3:** Data mining processing flow.

**Figure 4:** Architecture of data mining.

**Figure 5:** Statistics on the ratio of men to women and the number of injuries.

**Figure 6:** Example of knee injury.

**Figure 7:** Example of low back injury.

**Figure 8:** Occurrence of exercise injuries in different parts of the body.

**Figure 9:** Occurrence of different types of exercise injuries.

**Figure 10:** Exercise injury occurrence.

**Table 1:** Expert validity questionnaire survey.

Title	Number of people	*A*	*B*	*C*	*D*	*E*
Professor	6	2	2	2	0	0
Associate professor	4	2	1	1	0	0
Lecturer	2	1	1	0	0	0
Total	12	5	4	3	0	0

**Table 2:** Fitness motivation and exercise injury survey results.

	Health		Relieve work stress		Fat loss, shaping		Increase muscle mass	
	Male	Female	Male	Female	Male	Female	Male	Female
Total	49	47	20	7	10	58	65	0
Number of injuries	13	7	5	1	1	23	42	0
Aggregate injury rate	20.8%		22.2%		35.2%		64.6%	

**Table 3:** Nature and proportion of knee injuries.

Site and type of injury	Example	Proportion (%)
Knee sprain	5	27.2%
Knee joint strain	7	38.8%
Knee lacerations	4	22.2%
Other	2	11.1%

**Table 4:** Nature and proportion of lumbar injuries.

Site and type of injury	Example	Proportion (%)
Back sprain	9	37.5%
Low back strain	8	33.3%
Intervertebral disc injury	4	16.6%
Other	3	8.8%

**Table 5:** Health club exercisers sports injury causing factors statistics.

Sort by	Injury causing factors	Number of injuries	Percentage
1	Technical movements are not standard	12	11.2%
2	Unreasonable preparation activities	10	8.62%
3	Fatigue of the organism	9	7.76%
4	Excessive local load	8	6.89%
5	Against the principle of gradual and orderly progress	8	6.89%
6	Poor physical fitness	7	6.03%
7	Inattentiveness	7	6.03%
8	Coaching factors	7	6.03%
9	Excessive exercise load	6	5.17%
10	Venue and equipment factors	6	5.17%

## Data Availability

The data underlying the results presented in the study are available within the manuscript.
